RETRACTED

# Evaluation of College Students' IPE Environment Based on User Rating Sparsity and Big Data Technology

**DOI:** 10.1155/2022/3183195

**Published:** 2022-09-25

**Authors:** Nan Zou, Enfu Wang

**Affiliations:** YanShan University, Qinhuangdao 066004, China

## Abstract

Big data improves opportunities for enhancing and improving university students' IPE. In order to improve the accessibility of IPE for university students, this study integrates big-data techniques into the IPE (Ideological and Political Education) model of university students and builds the IPE platform. This study presents the idea of user rating sparsity and employs a two-step training strategy to address the issues of user cold start and sparse data in light of the drawbacks of conventional methods. This algorithm produces a very small data structure, which saves a lot of storage space. This study also uses hybrid recommendation technology, which effectively enables platform users to select customized update resources based on their interest information. According to test results, this method's suggestion accuracy can reach 95.69%, and it has a high user rating. This demonstrates that the method is reliable and accomplishes the desired result. This paper fully utilizes mega data to improve the accessibility of IPE for university students.

## 1. Introduction

Data has been in a state of continuous evolution in human life and keeps pace with the development of social phenomena [1]. It is one of the most concerned concepts in the information technology industry after the Internet of things and cloud computing. Big data contains valuable and useful information and value. The basic core development concept of big data is to analyze and integrate all data, and build a data management platform and data analysis model based on the integration of mega data samples [2]. This is fundamentally different from the traditional sampling survey and analysis in methodology and logic. Data is active in every corner of the campus. Whether it is the teaching process of students or their daily life, a great quantity of data message is constantly generated. How to filter and use these data message has become an important part of our education effect [3]. The analysis technology and mining technology in the Internet age have gradually received close attention from people. People in all walks of life have gradually realized that whoever has a deeper understanding of DM (Data Mining) [4] will seize the future opportunities. Therefore, in the Internet age, improving the availability of IPE for university students is no exception. Using big-data techniques to innovate IPECU (Ideological and Political Education in Colleges and Universities) is a brand-new topic. As a huge and complex information base, big data has high-end and cutting-edge technical characteristics. It is changing the way we observe the world and analyze and grasp problems around us in various ways. In the Internet age, the IPE of university students is affected by the environment and information technology, which makes the connotation of IPE change to a certain extent [5]. Big data is not only the carrier and tool of IPE but also runs through the instructional concept of IPE. The combination of the two constitutes a brand-new IPE method. Therefore, the big data IPE method is facing the dual innovation of development concept and development mode.

RETRACTED

IPE, in general, refers to social activities in which the society or social groups utilize particular ideologies, political viewpoints, and moral standards to control its members and shape them into ideological and moral figures that satisfy the interests of their own class [6]. IPE is a well-established practical activity, although its name and purpose have changed throughout time. University students are the country's new driving force, and their ideological framework has an impact on the way the whole country will evolve in the future. As a result, the IPE of university students is a very crucial role [7]. The goal of IPE for university students is to employ appropriate techniques to mentor and teach students in the new period, allowing them to grow into talents and develop in a healthy way. This establishes the theoretical basis for expanding the accessibility of IPE for university students. Although the big data development platform and concept are utilized, the emphasis is not on the technical level but rather on using big data into IPE strategies to enhance the effectiveness of IPE for university students. The application of big data can bring many opportunities for university students and educators, but there are also many challenges [8]. The details are as follows: ① The network information is mixed, good and bad, and the values of university students have not been fully established, so they are easily influenced by external information. ② In the process of data collection, there will inevitably be the risk of leakage, which will affect students' psychology. ③ At present, there are few professional technical talents in the field of big-data techniques, and most of the ideology educators lack relevant technologies, so the application of big data is not effective. Seize the opportunity to develop university students' IPE, effectively use big-data techniques to analyze and judge the development status of University Students' thoughts, psychology, and behavior, and constantly enhance the availability of university students' IPE [9].

RETRACTED

Based on this, this paper embeds big-data techniques into the analysis of college students' IPE mode, and its innovations are as follows:

1. This paper closely combines the characteristics of the current era and conforms to the theme of the current era; analyze the mode of IPE for university students by using today's big-data techniques. At the same time, it is closely combined with the current development practice of IPE and puts forward the innovation path of IPE in the Internet age
2. In view of the shortcomings of traditional algorithms, this paper introduces the concept of user score sparsity and uses a two-step training method to solve the problem of user cold start and sparse data

## 2. Related Work

Due to the continuous progress of cloud computing and AI technology, people gradually realize the advanced nature of big-data techniques, realize its great contribution to people, and have an important impact on all aspects of human social life. There are also some scholars who combine big-data techniques with IPE.

Rubén et al. started from the interpretation of the connotation and characteristics of big data and then studied the characteristics of IPECU in the Internet age and the value of improving the availability of IPE for university students in the Internet age [10]. Wang et al. summarized the opportunities and challenges faced by university students' IPE and teaching in the Internet age development [11]. Bennett et al. believe that the promotion of personalization of IPE for university students in the Internet age should not only make effective use of the favorable conditions created by big data but also fully consider the possible risks [12]. Samarakou et al. summarized the research methods of big data IPE and explained the development process of big data [13]. The problems arising from the integration of big data into university students' IPE are sorted out and summarized. LF et al. pointed out that further strengthening and improving the IPE of university students to achieve the purpose of effectively enhancing the availability of IPE of university students is a new goal and task faced by the ideology work of universities at present [14]. Mobbs et al. aimed at the challenges of big data in enhancing the availability of university students' IPE and discussed the countermeasures of big data for enhancing the availability of university students' IPE [15]. Weston et al. studied how to use Web mining technology and combine existing clustering technology to achieve high accuracy classification and clustering of Web text data [16]. Nurse et al. built an instructional resource recommendation system based on online education, and designed and implemented each module of the system; describe the development platform and tools, and test the actual development effect [17]. According to the fundamental data of resource users, Lee et al. used the customized service mechanism in the system and rule-based recommendation technology, which successfully achieved the personalized initial resource selection of new users of the information platform [18, 19]. Based on users' browsing histories, habits, and interests, this recommendation system suggests educational resources that users may find interesting.

RETRACTED

After defining the related concepts in the Internet age, this paper makes an in-depth summary and analysis of university students' thoughts, behaviors, and specific activities. At the same time, the innovation path of IPE in the Internet age is put forward, and the IPE platform based on big-data techniques is constructed. It can improve the education and teaching level of ideology theory courses.

## 3. Methodology

### 3.1. Concept, Characteristics, and Types of Big-Data Techniques

The Internet age is a digital era based on the collation, practice, and innovation of massive network data. Big data starts the process of quantitative research. In the Internet age, everything can be quantitatively analyzed and studied, which provides great convenience for the human research process [20]. On the application level, mega data refers to the collection and integration of large-scale data in a certain range of time by using new data collection and processing tools. In practical applications, many database users will put many data sets together, thus forming PB-level data volume [21]. It mainly reflects the large amount of data and the integrity of data. The variety of data is also an important feature of big data. Traditional data are mostly relational data. Structured data refers to data or a unified structure, which we call structured data. This kind of structured data is easy to store, process, and query, but the extraction of this kind of structured data does not consider the correlation of things and lacks the grasp of details, so the form is relatively simple. The processing method of this kind of data is simple and easy to manage, while the data growth is slow. Big data is generated quickly, so the processing speed is required to be fast. Because of the explosive growth of data, it is constantly updated, and the technology of processing data has to be constantly improved to extract useful data. The speed of data processing determines whether data users can successfully mine valuable information. Low value density refers to the fact that with the expansion of data scale, the value of unit data decreases due to the significant reduction of the role of data in practice. Only by integrating data can the real value of mega data be brought into play.

RETRACTED

Big data is not only a technical means but also a resource and wisdom. There is a direct correlation between data scale and DM, and data includes structured data. If there are big waves in these massive data, finding out the really valuable information is the real value of big data [22]. There are many ways to divide the types of big data. This paper only takes the data source as the boundary to distinguish the types of big data. Depending on different data sources, transaction data of data platform, historical data of interactive information platform, unstructured data of artificially constructed information system, etc. are all types of mega data. At present, it has entered the Internet age and has made important changes in the field of education. In the Internet age, the network environment has a great influence on IPECU. With the use of big-data techniques, the human spiritual world that was difficult to objectify and digitize in the past has become like the objective material world and can be described and recognized by data, which has brought the technical means to the research and practice of university students' IPE. Combined with the characteristics of mega data and IPE, the IPE in the Internet age can be defined as relying on the development platform of big data, using the ideas of data thinking, and using the educational methods and ideas in the era of data, trying to carry out the practice process of IPE. Value is the ultimate meaning of big data, which can help decision makers predict the development direction of things and realize scientific decision-making. The core of big data is prediction. As the core of big data forecasting, the decision-making and guidance of university students' IPE will have a good effect, and forecasting will help to improve the availability and pertinence of university students' IPE. In the education industry, the advantages gained by the application of big data will become more obvious, which will bring unprecedented important changes to education.

### 3.2. Innovation Path of IPE in the Internet Age

New technology and approaches have been introduced to university students' IPE by the Internet era. The traditional Chinese philosophy of “teaching students in accordance with their aptitude” and the theory of “interactive teaching” were the key influences on the big data instructional mode of IPECU in the past [23]. The significance of data permeates the entire IPE process, and the deliberate, planned, coordinated, and targeted influence is carried out by gathering member data in order to increase the scientific rigor and breadth of IPE. The use of appropriate techniques is essential to the goal of IPE. Utilizing rational, efficient, and effective strategies to better direct and teach university students is essential to the success of IPECU. The objectives and responsibilities of IPE must be continually clarified if its accessibility to university students in the Internet age is to be strengthened and improved. Utilize big data approaches to their maximum potential in order to achieve true tailored learning. According to the big data perspective, university students' ideology teachers must introduce the idea of big data and foster thinking that is flexible for the Internet era. Ideology instructors must learn DM technology and mine all student data if they want to develop new skills and methodologies. To establish the big data instructional mode of university students' ideology theory course, we should lay stress on the following application conditions and effectively improve the availability of education and teaching: ① Emphasize the use of modern digital technology. ② It needs to establish an instructional resource database. ③ It needs to introduce the double-subject instructional concept. ④ The instructional effect of instructional mode can be maintained and tracked for a long time. Innovating IPECU requires college teaching to keep pace with the development of the times. Educators should constantly improve their own knowledge connotation and instructional methods, focus on the personality characteristics and practical needs of university students, and promote the communication between educators and educatees. Use new knowledge and skills to improve the availability of IPE and the overall level of instructional quality and scientific research management in universities. At the same time, big data provides new technologies and new methods for university students' ideology personalized education, which will surely lead to profound changes in IPECU. Ideology educators should actively update their educational concepts and actively adapt to the development requirements of the new era.

RETRACTED

It is that primary task of chan the traditional education mode to carry out the predictive model of IPE and to establish the predictive thinking of educator. Prediction is to judge what will happen in the future, and the core function of big data is prediction. Ideology educators of university students have collected all the data of university students. After sorting and analyzing these data, educators should lay stress on the correlation of these data. The Internet age provides technical support for IPE, but it is often because educators do not lay stress on big data that it is difficult to integrate big data with IPE, so it becomes an obstacle to modernization. Therefore, it needs to improve educators' data thinking. Set up predictive thinking to solve students' problems by using data science. In the Internet age, university students' ideology educators can better grasp university students' ideological trends through in-depth analysis of massive data message, thus achieving better decision-making and management. In addition, the IPE environment outside the network makes the two sides who communicate with each other become reality. The two sides can not only exchange ideas and feelings but also realize the effective transmission of information, mutual learning, and mutual inspiration. In terms of teaching objectives, big data will inevitably produce quantitative results, which requires that when constructing the instructional mode of IPECU, data should be collected and analyzed first, so as to increase the supporting effect of data on teaching objectives. We should give full play to the persuasive role of big data and fully understand the ideological trends of university students. In terms of teaching philosophy, the sharing characteristics of big data require educators and educational objects to participate together, adopt the cooperative learning method, jointly explore the characteristic parts of data, and interpret and attribute them with empirical thinking. In addition, in order to make big-data techniques better used in university students' IPE practice, it is necessary for universities to vigorously cultivate corresponding big-data techniques capabilities among counselors, class teachers, ideology theory teachers, and other teams. The outstanding characteristics and advantages of the Internet age are massive data message and various forms of media. As the first duty subject of university students' IPE, only by grasping the core of big data management can we achieve effective results of IPE. The IPE in the Internet age focuses on the direction of data, trains students and educators to think about data, and replaces the traditional experiential teaching with more scientific intuition. In the process of gradual digitization, teachers' ideological work is more targeted, and students are better understood and targeted. The main position of the educational subject in the teaching process is also constantly highlighted, which stimulates the enthusiasm of educators. In terms of instructional methods, the rapid development of technology in the Internet age promotes the innovation of instructional methods. If dual-subject teaching is an idea, then schema teaching, video teaching, and dual-classroom teaching are the concrete methods to implement this teaching idea. The introduction of big data thinking into university students' IPE class ultimately requires updating the instructional methods to realize the practice of values and instructional concepts. The advent of the Internet age provides university students with a cognitive way to complement each other's knowledge and learn from each other. Undeniably, the Internet age has provided us with massive information resources, and most knowledge points can be obtained free of charge in the network. University students can use various online learning platforms to obtain massive knowledge, massive information, and massive resources, which is diverse for university students to acquire knowledge.

RETRACTED

The fundamental task of IPE when using big data to create predictions is data gathering and processing. The direction that instructors give to students' education will be impacted by inappropriate data collecting, incomplete receipt collection, wrong data processing, and inaccurate projections. As a result, data processing and gathering are crucial, and schools should pay attention to them. In the era of the Internet, we can better forecast the IPE of university students and finally actualize the trend of intelligent development by gathering vast amounts of data from university students and assessing the potential values and internal laws among these facts. Additionally, by creating a big data platform for IPECU and enhancing the capability of gathering, storing, and evaluating data, even feelings and thoughts that were previously believed to be challenging to quantify can overcome the limitations of conventional educational methods and ideas in the past and achieve quantitative research. The use of big data approaches offers technical assistance for IPE across the board. The accomplishment of all-staff education, whole-process education, and all-around education is supported by the integration of social resources with higher education resources. In order to increase the impact of IPE, network teaching should be done in conjunction with traditional education. Big data is required to enhance and innovate IPECU's teaching methodology, as shown by the teaching assistants and educational philosophy of today. It can only fulfil its proper job by developing a fair mode. In general, big data application instructors should accurately understand the benefits that big data techniques bring, work to increase their awareness of big data applications, and learn big data skills; being adept at utilizing big data thinking to develop and address relevant issues; utilize the benefits of big data to their fullest, improve IPE accessibility for college students, and constantly develop new IPE techniques.

RETRACTED

### 3.3. Construction of IPE Platform Based on Big-Data Techniques

The information mining module is the key component to establish this intelligent and personalized teaching environment. It mainly uses DM technology to analyze the data in the database, recommend the learning content to learners, and provide teachers and administrators with relevant mining patterns and rules. The platform structure mainly includes three parts, namely, student client, teacher client, and administrator client. At the same time, the teaching activities are divided into three modules: before, during, and after class. In the three modules, teachers, students, and administrators have different functions, and each function corresponds to a different learning task. The system administrator is mainly responsible for the management of system user information and operation rights. At the same time, he reviews the instructional modes imported into the system and performs related operations such as classification, label setting, and resource description, providing initial static attribute data of resources for later model building, DM, and recommendation. The platform has two main functions: ① Collecting information of students' learning behavior. ② Present the learning content recommended by the learning scheduling system. The platform provides the management interface of instructional resource database and teaching strategy database. At the same time, the analysis information obtained by the mining module is presented. The data collection module is the foundation of personalized teaching on the platform, and the type of data collected is established by the user analysis model of personalized network instructional platform. This is the data source of personality analysis engine, and the quality and quantity of collected information will directly affect the quality of personality system analysis. The information acquisition module is responsible for collecting the information and sending it to the next data processing module. The data flow diagram of resource-related functional modules is shown in Figure 1.

PageRank basically measures how important a page is, how many links point to it, how important the pages that point to it are, or a combination of the three. As a starting point, consider the following:

(1) $$\begin{array}{c} PR\left(q\right)=\underset{\left(p,q\right)\in E}{\sum }\frac{PR\left(p\right)}{N_{p}}. \end{array}$$

Among them, *N*_*p*_ represents the out-degree of node *P*. To ensure the convergence of the iterative process, *M* must satisfy two conditions: one is that the directed graph *G* must be strongly connected; the other is that *M* must be acyclic.

(2) $$\begin{array}{c} M^{\prime }=cM+\left(1-c\right){\left[\frac{1}{N}\right]}_{N\times N}. \end{array}$$

Using *M*′ instead of *M* for operation is equivalent to adding two edges between every two nodes of *G*. Additionally, doing so resolves the Rank Sink problem, whose iterative form is as follows:

(3) $$\begin{array}{c} {PR}_{i+1}=cM\times {PR}_{1}+\left(1-c\right)\times {\left[\frac{1}{N}\right]}_{N\times 1}. \end{array}$$

In this way, in the case of ensuring the convergence of iterations, the definition of PageRank is also changed to: let page *T*_1_, *T*_2_ ⋯ *T*_*n*_ have links pointing to page *A*:

(4) $$\begin{array}{c} PR\left(A\right)=\left(1-c\right)+c\left[\frac{PR\left(T_{1}\right)}{N_{T_{1}}}+\cdots +\frac{PR\left(T_{n}\right)}{N_{T_{n}}}\right]. \end{array}$$

Equation (4) is the PageRank iteration formula.

RETRACTED

In the system, there are many equal resource distribution centers in different geographical locations, and each center can independently provide personalized distribution services to resource users. This not only effectively solves the bottleneck problem of centralized and hierarchical server load but also does not increase the burden of resource users like the mesh type. In addition, this paper divides the index vocabulary into two parts. The former part is the words in common dictionaries. These terms are fixed in length and the total number is certain, which is called a static dictionary. The latter part is the words that do not appear in the dictionary through the identification of unknown words, which is called corpus-based dictionary. In this paper, statistical methods are used to filter unlisted words. Instructional resource database is a collection of teaching contents, taking courses and knowledge points as units, and adopting tree-graph structure to organize data. It includes the knowledge related to IPE and the actual instructional resources. It consists of four parts: curriculum, curriculum units, knowledge points, and instructional resources. Users can create a data source for a relational database or data warehouse by selecting the Data Source Wizard function. For personalized service system, the most important thing is the participation of users, so in order to track users' interests and behaviors, this paper establishes a user model for each user. User model depicts the characteristics of users and the relationship between users. The use case diagram of recommendation function demand of IPE resources is shown in Figure 2.

In all user sets *C*, the idea of *k* nearest neighbors is adopted to find *k* users with the most similar preferences to the current user *c* to form the neighbor user set *C*′; then, according to the comprehensive score of the neighbor user set *C*′ on the resource *s*, the current user *c* pair is predicted Resource *s* preferences. The similarity between users is measured by their common rating items, which are often calculated by the Pearson correlation, namely:

(5) $$\begin{array}{c} \text{sim}\left(c_{i},c_{j}\right)=\frac{\sum_{S\in I_{ij}}\left(R_{i,s}-\bar{R_{i}}\right)\left(R_{j,s}-\bar{R_{j}}\right)}{\sqrt{\sum_{S\in I_{ij}}{\left(R_{i,s}-\bar{R_{i}}\right)}^{2}}\sqrt{\sum_{S\in I_{ij}}{\left(R_{j,s}-\bar{R_{j}}\right)}^{2}}}. \end{array}$$

Among them, *I*_*ij*_ represents the common scoring resource set of users *c*_*i*_ and *c*_*j*_; *R*_*i*,*s*_ and *R*_*js*_ are the resource ratings *s* of users *c*_*i*_ and *c*_*j*_; $\bar{R_{i}}$ and $\bar{R_{j}}$ are the average scores of users *c*_*i*_ and *c*_*j*_ to the rated resources. The more similar the ratings of the common rating items, the greater the Pearson correlation value, indicating the greater the similarity between users.

RETRACTED

After obtaining the nearest neighbor user set *C*′ of the current user *c*, the resource *s* is scored and predicted, that is:

(6) $$\begin{array}{c} P_{c,s}=\bar{R_{c}}+\frac{\sum_{e\in C^{\prime }}\text{s}\text{im}\left(c,e\right)\times \left(R_{e,s}-\bar{R}e\right)}{\sum_{e\in C^{\prime }}\left|\text{sim}\left(c,e\right)\right|}. \end{array}$$

Among them, sim(*c*, *e*) represents the similarity between user *c* and user *e*; *R*_*e*,*s*_ is the score of resource *s* by user *e*, and $\bar{R_{c}}$ and $\bar{R_{e}}$ are the average scores of users *c* and *e* on the rated resources.

When the rating matrix is sparse, there are few resources shared by two users, but their similarity may be high. Therefore, this paper introduces the concept of user rating sparsity, which is equal to the ratio of the number of common comment resources of users *u*_1_ and *u*_2_ to the union of the two user comment resources, as shown in Formula (7):

(7) $$\begin{array}{c} {\text{sparsity}}_{u_{1},u_{2}}=\frac{\left|I_{u_{1}}\cap I_{u_{2}}\right|}{\left|I_{u_{1}}\cup I_{u_{2}}\right|}. \end{array}$$

Similarly, the score sparsity of resources *i*_1_ and *i*_2_ can be expressed as Equation (8):

(8) $$\begin{array}{c} {\text{sparsity}}_{i_{1},i_{2}}=\frac{\left|U_{i_{1}}\cap U_{i_{2}}\right|}{\left|U_{i_{1}}\cup U_{i_{2}}\right|}. \end{array}$$

If the characteristic attribute vector of resource *i*_1_ is:

(9) $$\begin{array}{c} {\overset{⟶}{l}}_{1}=\left\{C_{11},C_{12},\cdots ,C_{1m}\right\}. \end{array}$$

The feature attribute vector of *i*_2_ is:

(10) $$\begin{array}{c} {\overset{⟶}{l}}_{2}=\left\{C_{21},C_{22},\cdots ,C_{2m}\right\}. \end{array}$$

Then, the similarity of feature attributes between two resources can be expressed as:

(11) $$\begin{array}{c} {\text{sim}}_{\text{Attr}}\left(i_{1},i_{2}\right)=\frac{{\overset{⟶}{l}}_{1}\cdot {\overset{⟶}{l}}_{2}}{\left\|{\overset{⟶}{l}}_{1}\right\|\cdot \left\|{\overset{⟶}{l}}_{2}\right\|}. \end{array}$$

Then, the similarity formula between two resources is:

(12) $$\begin{array}{c} {\text{sim}}^{\prime }\left(i_{1},i_{2}\right)=\alpha \cdot {\text{sparsity}}_{i_{1},i_{2}}\cdot {\text{sim}}_{R}\left(i_{1},i_{2}\right)+\left(1-\alpha \right)\cdot {\text{sim}}_{\text{Atrr}}\left(i_{1},i_{2}\right). \end{array}$$

Among them, sim_*R*_(*i*_1_, *i*_2_) is the similarity between two resources calculated according to the scoring matrix; *α* is the weight value. It can be seen from the above formula that when the resources *i*_1_ and *i*_2_ have few or even no common scoring users, their similarity can still be calculated, which overcomes the problem of sparse data to a certain extent.

RETRACTED

The resource attribute matrix, user browsing and downloading matrices, and user score matrices are the inputs for the suggested algorithm. To avoid the cold start issue brought on by freshly registered users and newly added instructional materials, the recommendation module currently only accepts the intrinsic attributes of educational resources as input. The platform can offer recommendations in two different ways. Active recommendation is one. For instance, the system actively suggests relevant resources when a user browses or downloads a resource. The other is passive suggestion, where the system passively suggests related information once the user selects the recommendation tab. This platform simultaneously offers students two very distinct learning strategies, one of which allows students to select their own knowledge material that they feel they have not understood well enough based on the course directory tree. The network instruction platform also automatically provides feedback and makes intelligent judgments and adjustments based on the students' responses as it systematically presents the explanation and test of knowledge points in accordance with the pre-set teaching content and teaching sequence of the corresponding target level. Through the use of natural language processing and semantic search, man-machine interfaces provide interactive features between the system and users. The interactive interface allows decision makers to input their instructions into the system and output DM outcomes, knowledge patterns from the knowledge base, and OLAP analysis results.

RETRACTED

## 4. Result Analysis and Discussion

After realizing the IPE platform based on big-data techniques, this section designs an evaluation experiment for the model to quantitatively get the performance index of the model. In this way, we can have a deeper understanding of the advantages and disadvantages of the model, and at the same time provide a reference for the optimization of model parameters and the further optimization of the model. The programming language of this paper is C#. # C language is a modern language and the most important programming language in .NET platform. Developers can use it to create a wide range of applications for the new .NET platform. # C programming language is easy to operate, powerful, object-oriented, and type-safe. The goal of C is to combine the high productivity of Visual Basic with the ability of C++ itself. The specific platform development environment is shown in Table 1.

The experimental data of this experiment is the training data of the homepage recommendation module collected from the user operation logs in this platform. When users log on to the platform, browsing, learning, or collecting courseware produces a series of learning behaviors, which are recorded in Web logs. By analyzing the Web log file, we can get the IP of the remote host used by the user, the access time, the specific Web resources browsed, and the request return code.  Figure 3 shows the training of the algorithm.

When the user visits the resource detail page and scores the instructional resources, the training data collection process recommended by the homepage will be triggered. This process will record the recommendation degree of this instructional resource and the scoring characteristic value of the user when the current user scores, and then save it in the database.  Figure 4 shows the precision comparison results of the algorithm.  Figure 5 shows the comparison of recall rate of the algorithm.

It can be seen that the precision and recall of this method are both excellent.

The resource display and learning module shows learners the instructional resources recommended by the recommendation method implementation module, and provides support functions such as learning and browsing, and collects learners' behavior information in real time. Users are mainly students and teachers. Students learn on the platform according to their own interests and personalized recommendation results. As the most important data source, students' achievement in IPE platform needs to be designed with emphasis, among which the student table and achievement table are shown in Table 2. The student client table and the teacher client table are shown in Table 3.

RETRACTED

The off-line experiment method is used to verify the correctness of the improved algorithm. Each experiment selects a subset, and the improved algorithm is used to predict the users' scores on the base data set. Then, the real scores of the test are used to calculate the error of the prediction scores to verify the availability of the algorithm. The *f* value of the algorithm on different data sets is shown in Figure 6.

The platform constructed in this paper is for teachers and students, so 300 teachers and 300 students are randomly selected to rate the resources recommended by different platforms.  Table 4 shows the evaluation of users' satisfaction with the resources recommended by different platforms.

The user's homepage suggestion module of educational resources will be trained based on the user's scoring behavior and the desired data after the model training module reads the user's scoring records from the database. The user's model will be saved after training. Finally, recommend instructional resources to users in accordance with the new recommendation degree after calculating the recommendation degree of ideology instructional resources based on the new user preference matrix. The recommended accuracy of different methods is shown in Figure 7.

This section makes an experiment on the platform and algorithm of IPE based on big-data techniques. The test results show that the recommendation accuracy of this method can reach 95.69%, and a high user rating is obtained. This shows that the algorithm has certain reliability and achieves the expected goal. With the increase of the number of learners and the accumulation of learning behaviors, the grading information of instructional resources gradually increases, the sparseness of the grading matrix decreases, and the quality of the improved algorithm is improved. So as to improve learners' learning interest and efficiency, promote more learners to enter the platform, and form a virtuous circle.

## 5. Conclusion

Big data provides a new way for human beings to know and transform the world, and it is a new tool and technology to promote the continuous development of society. Research on the availability of improving university students' IPE in the Internet age not only determines the safety of college ideological field but also closely links with university students' thinking orientation. In this paper, mega data is integrated into university students' IPE, so that educators can tap the potential value of student data, study the law of university students' thoughts and behaviors, help university students develop their world outlook, outlook on life and values, and realize their free and all-round development. In view of the shortcomings of traditional algorithms, this paper introduces the concept of user rating sparsity and uses two-step training method to solve the problem of user cold start and sparse data. The data structure generated by this algorithm is very compact, which saves a lot of storage space. Finally, this paper makes an experiment on the platform and algorithm of IPE based on big-data techniques. According to test results, this approach can produce recommendations with an accuracy of up to 95.69% and has a good user rating. This work proposes an improved approach that may efficiently reduce the sparsity of the scoring matrix and enhance the quality of the recommendation algorithm. This demonstrates that the algorithm is rather reliable and succeeds in achieving the desired outcome. In order to maximize IPE among university students and raise the bar, this paper makes extensive use of big-data approaches. Build a big data development platform-based interactive teaching (IPE) mechanism between professors and students in the new development environment to raise the caliber of instruction for courses in ideology theory.

RETRACTED

## Figures and Tables

**Figure 1:** Data flow diagram of resource-related functional modules.

**Figure 2:** Use case diagram of recommended function requirements for IPE resources.

**Figure 3:** Algorithm training situation.

**Figure 4:** Precision comparison results.

**Figure 5:** Comparison of recall results.

**Figure 6:** The *F* value of the algorithm in this paper on different data sets.

**Figure 7:** Recommendation accuracy of different methods.

**Table 1:** Platform development environment.

Exploitation environment	Set
Hardware environment	Pentium D CPU 2 8GHz, 1GB RAM
Operating system	Windows XP
Development platform	Microsoft ASP. Net
Web server	IIS
Programming language	C#
Database system	Access

**Table 2:** Student table and grade table.

Student		
1	Studet-NO	Char (20)
2	Studet-name	Varchar (20)
3	Studet-sex	Varchar (2)
4	Studet-age	Char (2)
5	Studet-collge	Varchar (20)
6	Studet-major	Varchar (35)

Transcript		
1	Student-NO	Char (20)
2	Class-NO	Char (10)
3	Achievement	Varchar (4)
4	Fail	Varchar (1)
5	Curriculum nature	Varchar (2)

**Table 3:** Student client table and teacher client table.

Student client		
1	Student-ID	Varchar (20)
2	Password	Char (30)

Teacher client		
1	Teacher-ID	Varchar (20)
2	Password	Char (30)
3	College-NO	Char (3)
4	Major-NO	Char (6)

**Table 4:** User satisfaction evaluation of recommended resources on different platforms.

Method	Teacher	Student
Based on user's recommendation	78.54%	79.21%
Content based recommendation	85.36%	86.11%
Project-based recommendation	87.24%	86.79%
Recommended method in this paper	94.87%	95.68%

RETRACTED

## Data Availability

The data used to support the findings of this study are available from the corresponding author upon request.
